This article has been retracted.

# Application of Wavelet in Quantitative Evaluation of Gait Events of Parkinson's Disease

**DOI:** 10.1155/2021/7199007

**Published:** 2021-12-09

**Authors:** Noore Zahra

**Affiliations:** College of Computer and Information Sciences, Princess Nourah bint Abdulrahman University, Riyadh, Saudi Arabia

## Abstract

**Results:**

Systems detected FOG and other gait postures and showed time-frequency range by examining differentiated decomposed signals by DWT. Energy distribution and PSD graph proved the accuracy of the system. Validation is done by the LOSO method which shows 90% accuracy for the proposed method.

**Conclusion:**

Observations of the clinical trials validate the proposed technique. In comparison to the previous techniques reported in literature, it is seen that the proposed method shows improvement in time and frequency resolution as well as processing time.

## 1. Introduction

Parkinson's disease (PD) is a neurogenerative disorder prevalent in persons above the age of 65 due to the loss of dopaminergic neurons in the basal ganglia [1]. This results in major cardinal movements like bradykinesia, stiffness, and distal tremor [2]. Besides this impairment, freezing is also the most common symptom. Freezing may lead to blocking of certain movements while walking due to the inability to generate effective stepping. Freezing of gait (FOG) is the reduction or episodic absence of the forward progression of feet due to which PD patients cannot move their feet leading to falling [3, 4]. According to a survey report, about 6620 patients are suffering from FOG [4–6].

Consequently, such patients have faced an inability to perform tasks of daily life, i.e., turning and gait initiation [4, 5].  Figure 1 shows different gait events involved in walking, FOG, and standing. In FOG event, patients try to move their legs to step forward but are unable to do so. The Hoehn and Yahr scale uses mostly five stages of PD symptoms according to the level of disability [7]. These are as follows:

- Unilateral involvement
- Bilateral involvement
- Bilateral disease
- Severe disability
- Wheelchair-bound

In unilateral involvement, one side of the body is affected while in bilateral both sides of the body are involved; however, the patient can move independently—no balance problem is observed. As the patient approaches, the third stage balance impairment is found. In the fourth stage, though the condition deteriorates, the patient can walk or stand without help. In wheelchair-bound condition, the patient is unable to stand or move unassisted and is bedridden in most cases.

PD affects the motor skill of the patient which leads to slowness and freezing of gait. Drug dosage and composition directly impact motor activity. However, determining the regimen of drugs has been a frequent problem which the clinicians face.

Gait assessment is an effective clinical tool to measure human locomotion. It may apply to the diagnosis of the medical condition of a PD patient. Clinical assessment and video analysis of lab activities are available as the tools to assess gait impairments. However, these depend on questionnaires (UPDRS), description ability of patients, and experience of clinicians. Hence, automatic detection of FOG is considered highly desirable [8]. The wearable sensor technologies have made it possible to assess FOG more intensively and objectively [9]. These wearable devices may be used for a long term to monitor patients as they are portable, comfortable, and lightweight.

Several attempts have been made to detect gait impairment using electroencephalogram (EEG), electromyograph (EMG), wearable sensors, etc. Nieuwboer et al. had tried to figure out lower limb muscle activity before freezing by analyzing temporal pattern and magnitude of electromyograph (EMG) [10]. Handojoseno et al. tried to predict the transition from walking to FOG using EEG [11]. Moore et al. in 2008 defined freeze index, which differentiates between freeze band and locomotion band [12]. Bachlin et al. detected FOG events online using wearable health assistants by providing Rhythmic Auditory Stimulation (RAS). They have taken 8 hours and 20 min of data from sensors among ten patients where eight exhibited FOG events. About 0-66 per-patient FOG events were identified. 95% of the FOG events are seen within the first 30 seconds of movement. The researchers have extracted five main statistical features from the sensors' signals [13]. In 2019, Guo et al. detected FOG and calculated FI using the Asymmetric Basis Function Time-Varying Auto-Regressive Moving Average Method (TV-ARMA). They first identified TV-ARMA then estimated parameters by transforming the TV-ARMA model into the frequency domain and calculated FI by estimating the time-frequency spectrum [14]. Li et al. in 2020 detected FOG by deep learning technique. They used 1-D deep convolution neural network for feature extraction; further, they introduced squeeze and excitation blocks to improve the detection performance [15]. Xu et al. used template matching methods for the detection of FOG [16] while Yu et al. did the quantitative analysis for posture instability and studied postural instability at early stages and direction-specific pattern for a decrease in stability [17].

Sensor-based monitoring is far effective, feasible, and economical than traditional methods. The acquired sensor data is processed and analyzed for motion classification, freezing of gait assessment, fall detection, etc.  Figure 2 shows a framework for monitoring devices which consist of a tiny computer or microcontroller as a processing unit to record data and online signal processing, sensors, memory card, batteries, and communication interfaces.

Wearable accelerometer is one of the most used sensors. It is wearable and attached to the patient's leg. Accuracy for the sensor's placement at ankles is about 94% for different postures, movements, and fall detection [1, 2]. The USB interface/Bluetooth link transmits the acquired data to a computer for signal processing, programming, etc. In addition, ZigBee and Wi-Fi can extend the system to enhance its applicability.

This paper attempts to differentiate between patients based on level of disability, which may help doctors prescribe dosage of levodopa and carbidopa according to the degree of slowness of pace and freezing of gait. Furthermore, the wavelet tool presented here will evaluate disease symptoms, which may indirectly support the evaluation of the dosage of drugs. The contribution of this work includes (1) signal processing of acceleration data, (2) analysis of the processed data using DWT and wavelet energy function, (3) detection of FOG and analysis of its accuracy of the proposed method, and (4) validation of result by the LOSO method.

## 2. Materials and Methods

Wavelet transform is a mathematical function capable of analyzing the changes of frequency content of signal over time. The wavelet transform decomposes a signal into frequency and scale. Some of its applications include manifesting and analyzing trends, patterns, fluctuations, discontinuities, and spikes according to scale. Wavelet transform utilizes variable-size windowing technique to break data into pieces, and its representation exhibits the resolution of different frequency components.

### 2.1. Wavelet

Wavelet is a function *ψ*(*t*) which once decomposed is expressed as (*ψ*_*a*,*b*_(*t*)) in form of scaling and translation [14].

(1) $$\begin{array}{c} \Psi_{a,b}\left(t\right)=\frac{1}{\sqrt{\left|a\right|}}\Psi \left(\frac{t-b}{a}\right), \end{array}$$

where *a* shows scale while *b* is translation with the condition:

- *a*, *b* ∈ *ℜ*
- *a* is nonzero

Let *f*(*t*) be a function where *f* ∈ *L*^2^(*ℜ*); then, the continuous wavelet transform (CWT) of the signal is defined as [14]

(2) $$\begin{array}{c} W\left(a,b\right)=C_{a,b}=\int_{-\infty }^{\infty }f\left(t\right)\frac{1}{\sqrt{\left|a\right|}}\psi^{*}\left(\frac{t-b}{a}\right)dt=<f,\psi_{a.b}> \end{array}$$

where <., .> indicates inner product and “∗” means complex conjugate. Discrete wavelet transform (DWT) is calculated by discretizing parameters *a* and *b* which help in analyzing high frequencies and low frequencies by passing original signal into high-pass filter and low-pass filter; as a consequence, computation time reduces significantly [18–20].

Taking *a* = 2^−*j*^, *b* = *k*2^−*j*^ with *j*, *k* ∈ *Z*. By substituting this in (1), we get

(3) $$\begin{array}{c} \Psi_{j,k}\left(t\right)=2\frac{j}{2}\Psi \left(2^{j}t-k\right). \end{array}$$

The DWT can be written as

(4) $$\begin{array}{c} d_{j,k}=\int_{-\infty }^{\infty }f\left(t\right)2^{\frac{j}{2}}\Psi \left(2^{j}t-k\right)dt=<f,\Psi_{t,k}> \end{array}$$

where *j* is scale and *k* is location.

DWT is effectively implemented by multiresolution scheme [21–24] Multiresolution decomposition of *f*(*t*) at level H is defined as

(5) $$\begin{array}{c} f\left(t\right)=\overset{\infty }{\underset{k=-\infty }{\sum }}a_{H,k}2^{-\frac{H}{2}}\phi \left(2^{-H}t-k\right)+\overset{H}{\underset{j=-\infty }{\sum }}\overset{+\infty }{\underset{k=-\infty }{\sum }}d_{j,k}2^{-\frac{j}{2}}\psi \left(2^{-j}t-k\right)=A_{H}\left(t\right)+\overset{H}{\underset{j=-\infty }{\sum }}D_{j}\left(t\right) \end{array}$$

*ψ*(*t*) is the mother wavelet, while *ϕ* is a companion function, called scaling function [22].

(6) $$\begin{array}{c} \phi_{j,k}\left(t\right)=2^{-j/2}\phi \left(2^{-j}t-k\right). \end{array}$$

 *ϕ*_*j*,*k*_(*t*) represents approximation or scaling version of the original function *ϕ*(*t*).*a*_*H*,*k*_ at level *H* and is defined as

(7) $$\begin{array}{c} a_{H,k}=<f,\varphi_{H,k}> \end{array}$$

(8) $$\begin{array}{c} f\left(t\right)=\overset{+\infty }{\underset{j=-\infty }{\sum }}\overset{+\infty }{\underset{k=-\infty }{\sum }}d_{j,k}2^{-\frac{j}{2}}\psi \left(2^{-j}t-k\right) \end{array}$$

Let signal length be denoted by “*N*” where *N* = 2^*M*^. Let *T*_*s*_ be the sampling time. After decomposition, coefficients will be calculated as

(9) $$\begin{array}{c} t_{j,k}=k2^{j}T_{s}\;\left(k=0\cdots ,2^{M-j}-1\right) \end{array}$$

where 1 ≤ *j* ≤ *M*.

The wavelet expansion for level *M* would be

(10) $$\begin{array}{c} f\left(t\right)=\overset{M}{\underset{j=1}{\sum }}\overset{2^{M-j}-1}{\underset{k=0}{\sum }}d_{j,k}2^{-\frac{j}{2}}\psi \left(2^{-j}t-k\right), \end{array}$$

where *k* starts from 0 since we assume, without loss of generality, that the signal starts from *t* = 0 s.

#### 2.1.1. Energy Computation

The energy associated with the family {Ψ_*j*,*k*_(*t*) = 2^*j*/2^Ψ(2^*j*^*t* − *k*)} is given by

(11) $$\begin{array}{c} E_{j,k}={\left|d_{j,k}\right|}^{2} \end{array}$$

At resolution *j*, the overall energy is

(12) $$\begin{array}{c} E_{j}=\overset{2^{M-j_{-1}}}{\underset{k=0}{\sum }}{\left|d_{j,k}\right|}^{2} \end{array}$$

The total energy for the entire signal is expressed as

(13) $$\begin{array}{c} E_{tot}=\overset{M}{\underset{j=1}{\sum }}\overset{2^{M-j_{-1}}}{\underset{k=0}{\sum }}{\left|d_{j,k}\right|}^{2} \end{array}$$

At scale *j*, the coefficients are placed at instants *k*2^*j*^*T*_*s*_,*k* = 0, ⋯, 2^*M*−*j*^ − 1.

#### 2.1.2. Grouping and Spreading Out Energy

The signal will be divided into fixed-length windows where *L* = 2^*J*^*T*_*s*_.

Here, 2^*J*^ is the number of signal samples in the window.

Energy will be computed for each window at every resolution level *j*.

There are two cases taken under consideration:

Case (a) *J* > *j*: for this case, the window *n* : (*n* = 0, 1, ⋯, *N*_*W*_ − 1) have 2^*J*−*j*^ number of coefficients. Energy can be computed by grouping all the energy coefficients associated with the window:

(14) $$\begin{array}{c} \begin{array}{cc} {\hat{E}}_{j,n}=\underset{k}{\sum }E_{j,k} & \left\{\begin{array}{c} 0\leq k\leq 2^{J-j-1}-1,n=0\\ \left(2n-1\right)2^{J-j-1}\leq k\leq \left(2n+1\right)2^{J-j-1}-1,n=1,\cdots ,2^{M-J}-1 \end{array}\right. \end{array} \end{array}$$

Case (b) *j* > *J*: energy coefficients for scale *j* > *J* can be used:

(15) $$\begin{array}{c} {\hat{E}}_{j,n}=\frac{E_{j,k}}{2^{j-J}},k=\text{round}\left(\frac{n}{2^{j-J}}\right),\;n=0,\cdots ,2^{M-J}-1, \end{array}$$

round (*x*) rounds *x* to the nearest integer.

Total energy obtained for window *n* is

(16) $$\begin{array}{c} {\hat{E}}_{\text{tot},n}=\overset{M}{\underset{j=1}{\sum }}{\hat{E}}_{j,n}, \end{array}$$

and the relative energy for window *n* at resolution *j* is

(17) $$\begin{array}{c} {\hat{\rho }}_{j,n}=\frac{{\hat{E}}_{j,n}}{{\hat{E}}_{\text{tot},n}}. \end{array}$$

#### 2.1.3. Averaging Energy Coefficients

Moving average energy can be calculated as

(18) $$\begin{array}{c} \begin{array}{ccc} E_{j,n}=\frac{1}{2^{J-j}}\underset{k}{\sum }\underset{j,k}{\sum } & 0\leq k\leq 2^{J-j}-1 & n=0 \end{array} \end{array}$$

Total energy obtained for window *n* is

(19) $$\begin{array}{c} {\overset{¯}{E}}_{\text{tot},n}=\overset{M}{\underset{j=1}{\sum }}{\overset{¯}{E}}_{j,n},\;\text{ fo}r\;n\left(n=0,1,\cdots ,2^{M}-2^{J}\right), \end{array}$$

and the relative mean energy for the window *n* at resolution *j* is

(20) $$\begin{array}{c} {\hat{\rho }}_{j,n}=\frac{{\overset{¯}{E}}_{j,n}}{{\overset{¯}{E}}_{\text{tot},n}}. \end{array}$$

In the present work, the energy redistribution feature is used to identify FOG and differentiate between different gaits and for the evaluation of FOG quantitatively from the data obtained from the sensors attached to the body. Furthermore, it is shown that the different scales of decomposed wavelet show changes in the distribution of energy of the FOG data for different events of slowness, walking, standing, and freezing of gaits.

### 2.2. Gait Detection Algorithm

The patient's movement is measured by acceleration sensors which are placed on the shank, ankle, and thigh [13]. For this study, only shank data has been used for its strong motion signal characteristic which is better suited for the detection of FOG [15]. Measurement is presented in terms of the frequency component of these movements. FOG, walking, and standing gait are detected by analyzing these frequencies using wavelet transform. The data source in this paper is the UCI machine learning repository (Daphnet data) which is recorded from ten patients for more than 8 hours per patient. Data has been sampled at 64 Hz and signal length, *N* = 3000 with the time frame being 0.5 s. Wavelet function with Symlet wavelet is applied to discrete signals for decomposition. Number of decomposition level *M* = 6. DWT is applied for obtaining the approximation and detailed coefficients. After decomposition, the locomotion band (0.5 and 3 Hz) and FOG band (3 and 8 Hz) have been detected. The energy at every level for each data has been computed; then, the moving average is computed, which gives the energy thresholding limit. In the last step, detection of FOG, standing, and walking is done based on the distribution of energy. The algorithm for gait detection is given in the following.

Step1. Data acquisition from the body motion (through accelerometer).

Step 2. Preprocessing the data.

Step 3. Applying DWT on the data.

Step 4. Energy computation at each level.

Step 5. Energy averaging and thresholding.

Step 6. Detection of gaits (standing, walking, and FOG).

## 3. Results

### 3.1. Dataset

The Daphnet UCS repository dataset is a public dataset of 8 hours per patient of inertial signal data from 10 PD patients of the age group 59 to 75 years. These datasets were taken from acceleration sensors placed on the left thigh, the left calf, and the patient's back during performance of daily activities like walking and opening doors. The dataset used in this study was created by Bachlin et al. [13].

### 3.2. Application on Data Segments

The dataset has accelerometer signals for ten subjects. 20 s data has been taken from each subject's data, and FOG is seen in 3 subjects. The results were compared with the previous proved results shown in the literature [13] to validate the algorithm. Wavelet transform estimates the time of freezing event. In the first step, the signal has been split into smaller parts, and for these small pieces, transformation is calculated. After preprocessing the input signal, DWT has been applied to the input accelerometer signal, and the procedure is continued until the computation of the DWT coefficient reached at level 6. Coefficients of each level are plotted in the DWT plot; after each level of decomposition, a number of samples decrease. It is known that fewer samples are used at low frequencies as the frequency decreases, time resolution decreases, and frequency resolution increases. DWT on acceleration sensor data which is sampled at 64 Hz has been illustrated. The first level corresponds to (16-32) Hz, and the next level corresponds to (8-16) Hz, and the subsequent levels being (4-8) Hz, (2-4) Hz, and (1-2) Hz with the final level corresponding to (0.5-1) Hz. It is observed from the decomposition plot; no significant information is available. The useful information is obtained between 3^rd^ and 6^th^ level. Among the ten subjects, walking, standing, and FOG episodes can be seen. Symlet 4 is chosen as the mother wavelet by hit and trial among different mother wavelets due to its accurate detection performance. Additionally, the order of the wavelet, i.e., length of window chosen as 4, improves the calculation of time-frequency spectrum without leakage.

Time-frequency spectra are shown in Figure 3 calculated by wavelet transform (WT). WT is able to show time-frequency transient features that will help in detecting different gaits and FOG.

### 3.3. Energy Computation

The analysis of acceleration signal has been done based on the following computations: after the decomposition of signal, computation of the approximate and detailed coefficients is done using wavelet function “Symlet 4.” The coefficients so obtained are as follows: cD1-cD6, cA6. After computing these coefficients, energy has been calculated. Following are the results of the energy distribution and approximation. Level 6 has been chosen because with the further increase in the decomposition level, no significant information is obtained, i.e., at further transfer of energy into higher level beyond 6th level, the same pattern is obtained.

The proposed algorithm has been applied, and energy has been calculated for all the available data. Approximately similar results were obtained for same gait events, i.e., for FOG data, same type of energy distribution was obtained. To understand the analysis more clearly and conveniently, one case of a normal walk, one of standing, and one of FOG have been taken for discussion.  Table 1 represents energy distribution for signal pertaining to FOG, Table 2 pertaining to standing, and Table 3 corresponds to walking.

Figure 4 shows that in FOG, maximum energy is concentrated at the highest approximate level. About 3% of energy is at a detailed level where D1 corresponds to 1% of energy. In standing gait, about 60% of energy corresponds to approximate level, while the rest corresponds to detail level where D3 and D4 contain 13-14% of energy. In normal walking, there is about 80% of energy concentrated at the approximate level; there is a linear increase in detail levels.

In FOG and normal walk, maximum energy is concentrated at the level A6, while 1% of the energy for FOG and 2-5% for normal walk are concentrated at level D1, which corresponds to the low-frequency range of DWT. For the energy distribution for walking, energy at detail levels is higher as compared to the other two cases, while energy in approximate levels is lower. At level D6, 21% of energy is concentrated, corresponding to the high-frequency range of white noise. Therefore, the energy content of approximate level A6 for standing gait is lower than the corresponding levels of FOG and walking.

Figures 5(a)–5(c) show the Power Spectral Density (PSD) of signals pertaining to FOG, walking, and standing with a sampling rate of 256 Hz. Automatic detection of FOG is developed by measuring frequency components and the relative energy associated with it. Human movements mainly lie within the frequency range of 0-30 Hz as obtained through the accelerometers. About 90-96% of the energy falls in this range for walking. If there is no movement, for example, during standing of FOG, only noise is dominating the frequency spectrum below 0.5 Hz, in which approximately 10% of signal energy is distributed over the rest of the spectrum.

### 3.4. Performance Evaluation

Table 4 demonstrates the obtained results which are evaluated for eight subjects using LOSO. Subjects 4 and 10 are excluded from the study as they were not showing FOG or other clarity in gait. Sensitivity, specificity, Area Under Curve (AUC), and percentage error are calculated and marked as performance measure to evaluate the proposed method. It is observed from the result that six out of eight subjects show AUC greater than 0.90 and five out of eight show error less than 10%. This shows the credibility of the proposed model.

The comparison of obtained wavelet (DWT) with the STFT, TV-ARMA (with RLS), and TV-ARMA (with LROFR) methods reported in [14] for the sensitivity and specificity for the same dataset is shown in Table 5.

In real-time application, computational time contributes a major part in making decisions related to drug dosage and timing which directly affects the risk of falling. The computational time from previous studies [14] and proposed is compared in Table 6.

It is observed from the results shown in Table 6 that the proposed method is faster than other methods which are highly desirable in automatic detection of gaits and FOGs.

## 4. Conclusions

Human activity and body movements mostly lie between 0 and 30 Hz frequency range, below 15 Hz for gait and postures, as obtained through the accelerometers. The results show that for body movement (i.e., below 15 Hz), 90-96% of the energy is concentrated, while the rest of the energy which is approximately 10% of the total is distributed in the rest of the frequency range. Results shown in this paper explore the capabilities of wavelet energy function with its multiresolution properties. Furthermore, it shows different frequency localization for different gait events.

The paper demonstrates that the complete information of gait events can be found in the different multiresolution levels. Proper reconstruction can be possible with these levels without the loss of any information. With proper use of this decomposition, detection of transient is possible. The energy function allows the detection of different gait events. Results further show that there is a rearrangement of the relative energy of acceleration signal recording among different frequency bands which distinguish different gaits. It is shown that the energy distribution of the signal changes among the different scales of wavelet representation at standing, walking, and during the Fog.

The results pertaining to Power Spectral Density, energy distribution graph, performance evaluation, and computational time show that the proposed system has good detection capabilities and can be applied for the automation of gait detection in Parkinson's disease. The obtained result demonstrates that wavelet energy function and power spectra are efficient tools for human gait detection to improve the automatic diagnosis of PD. Evaluation of FOG detection is done by a leave-one-subject-out (LOSO) cross-validation. From evaluated results, it is marked that FOG detection performs well (approx. 90%) by the presented method.

A detailed study can be carried out in the future by making use of the data collected from sensors. Sensor signal data can be taken as input after preprocessing and interpolation for use in the signal processing module, where feature extraction and feature selection may be done. The analysis of the segments used in this study can be extended to the entire signal which may detect multiple FOG events in one signal. In the next step, symptom intensity may be predicted by using the data, which may lead to the ascertaining of the drug regimen and pre-FOG anticipatory treatment. A clinical assistance system can be designed by using sensor signals for the diagnostics and therapeutics for PD.

## Figures and Tables

**Figure 1:** (a) Shows walking event; (b) shows FOG event; (c) shows standing event.

**Figure 2:** Monitoring device.

**Figure 3:** Differentiated decomposed signal after applying DWT shows time-frequency range of (a) standing, (b) FOG, (c) walking, (d) standing, (e) standing, (f) standing, (g) FOG, (h) standing, (i) walking, (j) walking, (k) walking, and (l) FOG.

**Figure 4:** Energy distribution graph up to 6^th^ level for FOG, standing, and walking: (a) energy distribution for FOG; (b) energy distribution for standing; (c) energy distribution for walking; (d) cumulative energy distribution.

**Figure 5:** (a) (PSD) of signal (walking); (b) PSD of signal (FOG); (c) PSD (standing); (d) total power in the PSD (in %).

**Table 1:** Energy distribution computation for the DWT of frequency range of FOG.

Signal	Ea	Ed1	Ed2	Ed3	Ed4	Ed5	Ed6
S1	98.7948	1.2052					
	98.0566	1.1994	0.7440				
	97.6146	1.1880	0.7369	0.4605			
	97.4257	1.1658	0.7321	0.4519	0.2335		
	97.1709	1.1300	0.7009	0.4381	0.2264	0.3337	
	97.1257	1.0652	0.6607	0.4129	0.2134	0.3145	0.2076

**Table 2:** Energy distribution computation for the DWT of frequency range of standing.

Signal	Ea	Ed1	Ed2	Ed3	Ed4	Ed5	Ed6
S2	95.4468	4.5532					
	91.3153	4.5126	2.1721				
	91.1263	4.4355	2.1349	2.3033			
	89.3270	4.2992	2.0694	2.2325	2.0719		
	84.7907	4.0869	1.9672	2.1223	1.9696	5.0634	
	64.7802	3.6865	1.7744	1.9144	1.7766	4.5673	21.5005

**Table 3:** Energy distribution computation for the DWT of frequency range of walking.

Signal	Ea	Ed1	Ed2	Ed3	Ed4	Ed5	Ed6
S3	98.3518	1.6482					
	95.6368	1.5968	2.6775				
	93.9205	1.5041	2.6059	1.9695			
	91.3815	1.3503	2.3394	1.7680	3.1607		
	85.3562	1.1625	2.0141	1.5221	2.7211	7.2240	
	84.8562	6.8790	4.6966	1.7383	1.3781	0.2294	0.2225

**Table 4:** The result of sensitivity, specificity, AUC, and EER% of subjects 1, 2, 3, 5, 6, 7, 8, and 9. Subjects 4 and 10 have not been taken for study.

Subject	Sensitivity	Specificity	AUC	EER %
1	0.969	0.970	0.967	11.2
2	0.969	0.971	0.970	6.8
3	0.883	0.885	0.881	16.9
5	0.819	0.820	0.817	25.3
6	0.988	0.990	0.983	5.8
7	0.989	0.991	0.986	3.78
8	0.996	0.999	0.998	4.81
9	0.968	0.970	0.965	3.1
Overall	0.948	0.949	0.945	9.7

**Table 5:** Sensitivity and specificity comparison of DWT with different approaches.

Methods	STFT	TV-ARMA (with RLS)	TV-ARMA (with LROFR)	Wavelet (DWT)
Sensitivity	85.64	84.16	86.35	94.8
Specificity	58.45	61.06	66.36	94.9

**Table 6:** Computational time comparison of DWT with different approaches.

Methods	STFT	TV-ARMA (with RLS)	TV-ARMA (with LROFR)	Wavelet (DWT)
Computational time (s)	0.4587	0.4605	24.8363	0.1992

## Data Availability

The data used in this study is available at https://archive.ics.uci.edu.
